The article "Down-regulation of osteoprotegerin expression as a novel biomarker for colorectal carcinoma" was published in 2016. Journal: Oncotarget.

# Down-regulation of osteoprotegerin expression as a novel biomarker for colorectal carcinoma

**DOI:** 10.18632/oncotarget.7885

**Published:** 2016-03-03

**Authors:** Hyun-Soo Kim, Gun Yoon, Sung-Im Do, Sung-Joo Kim, Youn-Wha Kim

**Affiliations:** ^1^ Department of Pathology, Severance Hospital, Yonsei University College of Medicine, Seoul, Republic of Korea; ^2^ Department of Obstetrics and Gynecology, Pusan National University Yangsan Hospital, Pusan National University School of Medicine, Yangsan, Republic of Korea; ^3^ Department of Pathology, Kangbuk Samsung Hospital, Sungkyunkwan University School of Medicine, Seoul, Republic of Korea; ^4^ Department of Pathology, Asan Medical Center, University of Ulsan College of Medicine, Seoul, Republic of Korea; ^5^ Department of Pathology, Kyung Hee University School of Medicine, Seoul, Republic of Korea

**Keywords:** osteoprotegerin, down-regulation, colorectal carcinoma, promoter methylation

## Abstract

A better understanding of tumor biology is important in the identification of molecules that are down-regulated in malignancy and in determining their role in tumor suppression. The aim of this study was to analyze osteoprotegerin (OPG) expression in colorectal carcinoma (CRC) and to investigate the underlying mechanism for changes in the expression of OPG. OPG expression was assessed in CRC tissue samples and cell lines. The methylation status of the *OPG* promoter region was determined, and the effects of demethylation on OPG expression were analyzed. The effects of recombinant OPG (rOPG) administration on cellular functions were also investigated. Clinical and prognostic implications of OPG protein expression in CRC patients were analyzed. The CRC tissues and cells showed significantly lower OPG expression. Pyrosequencing of OPG-silenced CRC cells revealed that the *OPG* gene promoter was highly methylated. Treatment with demethylating agent significantly elevated *OPG* mRNA and protein expression. rOPG significantly decreased cell viability and MMP-2 and VEGF-A production in CRC cells. Reduced OPG immunoreactivity was associated with aggressive oncogenic behavior in CRC. Also, OPG expression was found to be an independent predictor of recurrent hepatic metastasis and independent prognostic factor for worse survival rates. We demonstrated that OPG silencing in CRC occurs through epigenetic repression, and is involved in the development and progression of CRC. Our data suggest that OPG is a novel prognostic biomarker and a new therapeutic target for the treatment of patients with CRC.

## INTRODUCTION

Colorectal carcinoma (CRC) is one of the most prevalent forms of malignant tumors worldwide, with over 600,000 CRC-related deaths occurring annually [1]. Despite major advances in surgical techniques and equipment, chemotherapy and radiation therapy, the prognosis for CRC patients remains poor because of distant metastasis and recurrence [2, 3]. Traditionally, the identification of patients at high risk of recurrence or distant metastasis has depended on pathological characteristics, such as depth of invasion, nodal metastasis, stage group and perforation or invasion of adjacent organs. However, the current tumor-node-metastasis (TNM) classification system is limited in that it cannot offer a prognosis for individual patients [4]. To improve the outcome of patients with CRC, it is crucial to identify cancer-related genes that can serve as predictive and prognostic biomarkers to individualize therapy.

Osteoprotegerin (OPG) is a member of the tumor necrosis factor (TNF) receptor superfamily. It has been shown that OPG is involved in the development and progression of human malignancies [5–14]. Three previous studies have reported on OPG expression and its role in CRC. Pettersen and colleagues [12] and De Toni and colleagues [7] observed the expression of *OPG* mRNA and proteins in CRC cell lines, Tsukamoto and colleagues [13] reported a significant correlation between OPG expression and aggressive behavior of CRC including depth of invasion and distant metastasis and worse survival rates; they identified OPG overexpression as an independent predictive factor for tumor recurrence. However, these studies did not elucidate the mechanism by which these changes in OPG expression occur. Moreover, Pettersen and colleagues [12] analyzed OPG expression only in CRC cell lines and not in a normal colonic epithelial cell line, raising questions about the meaning of the increase in OPG expression in the CRC cell lines. These issues were reinforced by a recent study by Lu and colleagues [10], where OPG expression in various cancer cell lines, including CRC and nasopharyngeal carcinoma cell lines, was significantly decreased, or remained undetected. They also showed that promoter hypermethylation of *OPG* gene promoter was involved in the down-regulation of OPG expression.

In this study, we investigated the expression of OPG in CRC tissue samples. To understand the mechanism underlying changes in OPG expression, we then investigated OPG expression in CRC cell lines before and after treatment with a demethylating agent, 5-aza-deoxycytidine (5-aza-CdR). We also analyzed the methylation status of the *OPG* gene promoter in CRC cell lines. We further examined the association of OPG protein expression with the clinicopathological characteristics and prognosis of patients with CRC. Our results indicated that promoter hypermethylation is a mechanism of OPG down-regulation in CRC, and that OPG is involved in the carcinogenesis and progression of CRC. We suggest that OPG is potentially useful as a prognostic biomarker in CRC.

## RESULTS

### OPG expression in CRC cell lines

Western blot revealed that OPG protein expression was significantly reduced in the CRC cell lines, SW620 and HCT 116, when compared with CCD 841 CoTr (Figure 1A). ELISA results confirmed the findings of Western blot (Figure 1B) and showed OPG concentrations in SW620 (470.09 pg/mL; *P* < 0.001) and HCT 116 (195.62 pg/mL; *P* < 0.001) were significantly lower than that in CCD 841 CoTr (3754.77 pg/mL). Consistent with these findings, SW620 (normalized expression ratio, 0.06) and HCT 116 (normalized expression ratio, < 0.001) cell lines showed significantly lower *OPG* mRNA expression than CCD 841 CoTr (primer set #1; *P* < 0.001, both). *OPG* mRNA was readily detected in CCD 841 CoTr, while it was negligible in HCT 116. These results were confirmed by PCR with another primer set (primer set #2; normalized expression ratio, SW620, 0.11; HCT 116, 0.008).

**Figure 1:** OPG expression in human normal colonic epithelial (CCD 841 CoTr) and CRC (SW620 and HCT 116) cell lines (**A**) Western blot for OPG. (**B**) OPG protein concentration analyzed by ELISA. SW620 (470.09 pg/mL) and HCT 116 (195.62 pg/mL) had significantly lower levels of OPG protein than CCD 841 CoTr (3754.77 pg/mL). (**C**) Normalized *OPG* mRNA expression ratio analyzed by quantitative real-time RT-PCR. Black bars, PCR using primer set #1; white bars, primer set #2. *P < 0.05 versus CCD 841 CoTr.

### Mechanisms contributing to reduced OPG expression in CRC

Lu and colleagues [10] found that OPG expression is absent in all nasopharyngeal carcinoma cell lines examined and is significantly down-regulated in various carcinoma cell lines. They also showed that this down-regulation is associated with hypermethylation of the *OPG* promoter. Based on their observations, we considered promoter hypermethylation to be a possible explanation for the reduced OPG expression observed in CRC. We analyzed the methylation patterns at three CpG sites (−186 CpG, −182 CpG, and −166 CpG) in the *OPG* promoter region (Figure 2A). SW620 and HCT 116 showed significantly higher degrees of promoter methylation than CCD 841 CoTr, indicating promoter methylation to be directly responsible for the reduced OPG expression (Figure 2B–2C). CCD 841 CoTr displayed almost no methylation at the three CpG sites, which were almost entirely methylated in HCT 116. The methylation frequencies of the three CpG sites in the different cell lines are shown in Table 1.

**Figure 2:** OPG down-regulation by promoter methylation and effects of 5-aza-CdR treatment on the frequency of promoter methylation and the expression of OPG in CRC cells (**A**) CpG islands and the transcription start site of OPG. (**B**) Typical pyrograms from the cell lines examined. Each gray shaded column indicates a CpG dinucleotide assayed. Percentage of methylation at that CpG dinucleotide is indicated above. Yellow-shaded boxes indicate internal bisulfite modification control assessments. Methylation frequencies are shown as the ratio of methylated CpG sites/total CpG sites. (**C**) Frequency of promoter methylation. *P < 0.05 versus CCD 841 CoTr. (**D**) Reduction in CpG methylation frequency in CRC cells by demethylation. Treatment with 5-aza-CdR significantly decreased methylation of three CpG islands in the *OPG* gene in CRC cells. *P < 0.05 versus pretreatment. (**E**) Restoration of *OPG* mRNA expression by demethylation. Treatment with 5-aza-CdR significantly elevated *OPG* mRNA expression in CRC cells. In particular, HCT 116 expressed little OPG at baseline, however, 5-aza-CdR induced *OPG* mRNA with 1697.5-fold increase in HCT 116, when compared with pretreatment. *P < 0.05 versus CCD 841 CoTr. (**F**) Western blot analysis revealed that OPG protein expression was increased in a dose-dependent manner.

**Table 1:** Methylation status of multiple CpG sites in the *OPG* promoter region in CRC and normal colonic epithelial cell lines

Cell line	Methylation (%)			*P*-value
	−186 CpG	−182 CpG	−166 CpG	
CCD 841 CoTr	0.0	2.3	4.1	
SW620	13.7	18.2	24.9	**0.008**
HCT 116	87.4	100.0	97.8	**< 0.001**

The results highlighted in bold represent statistically significant values (*P* < 0.05).

In addition, to investigate the possible effects of methylation on OPG down-regulation, we treated the cell lines with the demethylating agent 5-aza-CdR. 5-aza-CdR treatment induced a marked reduction in the methylation frequency of all the three CpG sites (Figure 2D). This reduction was associated with a significant restoration of *OPG* mRNA expression, a 1697.5-fold increase in HCT 116 and a 7.2-fold increase in SW620, when compared with pretreatment levels (Figure 2E). The restorative effect of 5-aza-CdR on OPG expression in HCT 116 was confirmed by Western blot, showing that OPG protein expression was increased in a dose-dependent manner (Figure 2F).

### Effect of recombinant OPG on cell viability, MMP-2 and VEGF in HCT 116 cells

We found OPG to be down-regulated in CRC cells, raising the possibility that re-expression of OPG might inhibit tumor growth. To clarify the functional role of OPG, we investigated the effect of rOPG on cell viability of CRC cells. HCT 116 cells were incubated with rOPG at the indicated concentrations, and cell viability was verified using MTT assay. As shown in Figure 3A, rOPG reduced cell viability in a dose-dependent manner. At a concentration of 5 μg/mL, cell viability decreased to 5%. We found no inhibition of growth in control bovine serum albumin-treated cells at any concentration. Moreover, we tested the effect of rOPG on the level of MMP-2 and VEGF-A by Western blot (Figure 3B). MMP-2 and VEGF-A production was significantly reduced at 5 μg/mL rOPG in HCT 116 cells, suggesting that rOPG influences cell viability, invasiveness and angiogenesis of HCT 116 cells.

**Figure 3:** Effects of rOPG on cell viability and the levels of MMP-2 and VEGF-A in HCT 116 cells (**A**) MTT assay revealed that rOPG significantly reduced cell viability in a dose-dependent manner. In particular, at a concentration of 5 μg/mL, cell viability decreased to 5%. (**B**) Western blot analysis revealed that after rOPG administration, MMP-2 and VEGF-A production were significantly reduced in HCT 116 cells.

### Down-regulation of OPG in human CRC tissues and cell lines

We investigated OPG protein expression in CRC and normal colonic tissue samples using immunohistochemical staining. OPG immunoreactivity was predominantly cytoplasmic, although faint nuclear staining was noted in a few cells. OPG was not detected in the extracellular matrix or connective tissues. Diffuse and moderate-to-strong OPG immunoreactivity was observed in all normal colonic tissue samples (117/117, 100.0%), while reduced OPG expression was observed in 80 of 117 (68.4%) tumor tissue samples. OPG expression was moderate in 31.6% (37/117), weak in 33.3% (39/117), and absent in 35.0% (41/117) of CRC samples (Figure 4A). OPG expression in CRC was significantly decreased, compared with that of normal colonic tissue samples (*P* < 0.001; Table 2).

**Figure 4:** OPG protein and mRNA expression in CRC tissue samples (**A**) Cytoplasmic OPG immunoreactivity in normal colonic mucosa and CRC. (a) Moderate staining in normal colonic epithelial cells. (b) Moderate, (c) weak, and (d) negative staining in CRC cells. (**B**) *OPG* mRNA expression in matched normal and cancer tissue samples. Twenty-two of 30 CRC tissue samples exhibited significantly lower *OPG* mRNA levels than the matched normal colonic mucosal samples.

**Table 2:** OPG immunoreactivity in 117 CRC and normal colonic tissue samples

Tissue sample	Number of cases (%)				*P*-value
	Reduced		Preserved		
	0 (negative)	1+ (weak)	2+ (moderate)	3+ (strong)	
Normal	0 (0.0)	0 (0.0)	21 (17.9)	96 (82.1)	< **0.001**
CRC	41 (35.0)	39 (33.3)	37 (31.6)	0 (0.0)

The results highlighted in bold represent statistically significant values (*P* < 0.05).

We also assessed the levels of *OPG* mRNA in 30 fresh-frozen CRC tissue samples and their normal counterparts. We identified 22 (73.3%) CRC tissue samples with significantly lower *OPG* mRNA levels than the matched normal colonic mucosal samples (Figure 4B). This finding was consistent with the immunostaining results. The mean relative *OPG* mRNA expression ratios were 0.36 ± 0.05 in CRC and 1.00 ± 0.02 in normal colonic mucosa. The difference between the two means was significant (*P* < 0.001).

### Association of OPG immunoreactivity with clinicopathological characteristics of CRC

The correlations between OPG expression and the clinicopathological characteristics of CRC patients are presented in Table 3. We observed significant inverse associations between OPG expression and primary tumor size (*P* = 0.001), metastatic tumor size (*P* = 0.001), histological grade (*P* < 0.001), presence of nodal (*P* = 0.001) and hepatic (*P* < 0.001) metastases, occurrence of recurrent hepatic metastasis (*P* = 0.043), stage group (*P* = 0.003), and vascular invasion (*P* = 0.009).

**Table 3:** Correlation between OPG expression and clinicopathological characteristics of patients with CRC

Characteristics	Number of cases (%)		*P*-value
	Reduced	Preserved	
Age (years)			
≥ 61	41 (68.3)	19 (31.7)	0.992
< 61	39 (68.4)	18 (31.6)	
Gender			
Man	54 (70.1)	23 (29.9)	0.571
Woman	26 (65.0)	14 (35.0)	
Size of primary tumor			
≥ 5 cm	52 (82.5)	11 (17.5)	**0.001**
< 5 cm	28 (51.9)	26 (48.1)	
Size of metastatic tumor			
≥ 3 cm	31 (100.0)	0 (0.0)	**0.001**
< 3 cm	26 (70.3)	11 (29.7)	
Histologic grade			
3	3 (100.0)	0 (0.0)	**< 0.001**
2	72 (73.5)	26 (26.5)	
1	5 (31.3)	11 (68.8)	
Pathological tumor stage			
pT4	11 (91.7)	1 (8.3)	0.100
pT3	69 (65.7)	36 (34.3)	
Nodal metastasis			
Present	42 (85.7)	7 (14.3)	**0.001**
Absent	38 (55.9)	30 (44.1)	
First hepatic metastasis			
Present	57 (83.8)	11 (16.2)	**< 0.001**
Absent	23 (46.9)	26 (53.1)	
Recurrent hepatic metastasis			
Present	40 (90.9)	4 (9.1)	**0.043**
Absent	17 (70.8)	7 (29.2)	
Stage group			
IV	31 (77.5)	9 (22.5)	**0.003**
III	19 (100.0)	0 (0.0)	
II	30 (51.7)	28 (48.3)	
Lymphatic invasion			
Present	22 (81.5)	5 (18.5)	0.105
Absent	58 (64.4)	32 (35.6)	
Vascular invasion			
Present	12 (100.0)	0 (0.0)	**0.009**
Absent	68 (64.8)	37 (35.2)	

The results highlighted in bold represent statistically significant values (*P* < 0.05).

### Predictive value of OPG expression in recurrent hepatic metastasis

The presence of nodal metastasis (*P* = 0.015) and vascular invasion (*P* = 0.045), multiplicity (*P* = 0.001) of metastatic tumors, and reduced OPG expression (*P* = 0.043) were associated with recurrence of hepatic metastasis (Table 4). When these covariates were analyzed using multivariate logistic regression analysis, nodal metastasis (*P* = 0.018), multiplicity of metastatic tumors (*P* = 0.001), and OPG expression (*P* = 0.015) independently predicted recurrent hepatic metastasis. Reduction in OPG expression had a higher relative risk of recurrent hepatic metastasis (5.328) than nodal metastasis (4.405). In addition, the subgroup of node-positive/multiple hepatic metastases/OPG-reduced patients, obtained as a combination of the three independent predictors, had the greatest probability of developing recurrent hepatic metastasis (94%; Table 5). The probability of developing metastatic recurrence in patients in the node-negative/single hepatic metastasis/OPG-reduced subgroup (39%) was also higher than that for patients in the node-negative/single hepatic metastasis/OPG-positive subgroup (11%). Node-positive patients with a single hepatic metastasis were divided into two subgroups based on OPG level. Patients with reduced OPG expression had a higher probability of developing recurrent hepatic metastasis (75%) than patients with positive OPG expression (25%). Similarly, the node-negative/multiple hepatic metastases/OPG-reduced subgroup had a higher probability of developing recurrent hepatic metastasis (83%) compared to the node-negative/multiple hepatic metastases/OPG-positive subgroup (72%).

**Table 4:** Independent predictors of recurrent hepatic metastasis determined by multivariate logistic regression analysis

Characteristics	*P*-value for recurrent hepatic metastasis		Relative risk
	Univariate	Multivariate	
OPG expression			
Reduced/Preserved	**0.043**	**0.015**	5.328
Nodal metastasis			
Present/Absent	**0.015**	**0.018**	4.405
Vascular invasion			
Present/Absent	**0.045**	0.369	2.858
HCM multiplicity			
Multiple/Single	**0.001**	**0.001**	8.905

Statistically significant characteristics are shown.

The results highlighted in bold represent statistically significant values (*P* < 0.05).

**Table 5:** The probability of developing recurrent hepatic metastasis by analysis of a combination of independent predictive characteristics

Characteristics			Probability of recurrent hepatic metastasis
Nodal metastasis	Multiplicity of hepatic metastasis	OPG expression	
Present	Multiple	Reduced	0.94
Absent	Multiple	Reduced	0.83
Present	Multiple	Preserved	0.81
Present	Single	Reduced	0.75
Absent	Multiple	Preserved	0.72
Absent	Single	Reduced	0.39
Present	Single	Preserved	0.25
Absent	Single	Preserved	0.11

### Prognostic value of OPG expression in CRC

We determined the possible prognostic value of OPG for CRC using clinical follow-up information for the 117 patients. Univariate analysis for survival showed that presence of nodal metastasis (*P* = 0.002), recurrence of hepatic metastasis (*P* = 0.005), higher stage group (*P* < 0.001), presence of lymphatic (*P* < 0.001) and/or vascular invasion (*P* < 0.001), multiplicity of metastatic tumors (*P* < 0.001), and reduced OPG expression (*P* = 0.016) were significant predictors of poor prognosis (Table 5). The median survival time for patients with reduced OPG expression was 35 months, compared to > 10 years in patients with positive OPG expression (Figure 5). Patients with OPG-positive CRC had stable survival rates of 93.2% between two and four years after surgery and 76.6% after four years, as shown by Kaplan-Meier plots. In contrast, CRC patients with reduced OPG expression displayed a steady decline in survival during the observation period. Survival rates were 89.2% for 1 year, 63.9% for 3 years and 53.0% for 5 years in patients with OPG-reduced CRC, and 100.0% for 1 year, 81.4% for 3 years and 76.5% for 5 years in patients with OPG-positive CRC.

**Figure 5:** Kaplan-Meier plot for OPG expression in 117 patients with CRC Solid line, patients with OPG-reduced CRC; dotted line, patients with OPG-preserved CRC. Overall survival rate was significantly lower in patients with reduced OPG than patients with preserved OPG (*P* = 0.006). Median survival time was 35 months for patients with reduced OPG expression, compared with > 10 years for patients with preserved OPG expression.

We also conducted multivariate survival analysis using a Cox proportional hazard regression model. OPG expression, recurrent hepatic metastasis, stage group, lymphatic invasion and vascular invasion were independent prognostic factors influencing survival (Table 6). Nodal metastasis and multiplicity of metastatic tumors did not affect survival. This analysis demonstrated that reduced OPG expression in patients with CRC was associated with a significant hazard ratio of 3.132, comparable to the risk associated with stage group (3.245).

**Table 6:** Factors predicting worse survival of patients with CRC

Characteristics	*P*-value for survival		Hazard ratio
	Univariate	Multivariate	
OPG expression			
Reduced/Preserved	**0.006**	**0.022**	3.132
Nodal metastasis			
Present/Absent	**0.002**	0.066	2.020
Recurrent HCM			
Present/Absent	**0.005**	**0.011**	4.221
Stage group			
IV/III/II	**< 0.001**	**0.036**	3.245
Lymphatic invasion			
Present/Absent	**< 0.001**	**0.008**	2.918
Vascular invasion			
Present/Absent	**< 0.001**	**0.013**	2.666
HCM multiplicity			
Multiple/Single	**0.016**	0.072	2.243

Statistically significant characteristics are shown.

The results highlighted in bold represent statistically significant values (*P* < 0.05).

## DISCUSSION

Selecting the most beneficial treatment regimen for CRC remains challenging because of the lack of prognostic biomarkers [15]. We analyzed the expression of OPG in human CRC tissue samples and found that 73.3% of samples had significantly reduced *OPG* mRNA expression and 68.4% had significantly reduced protein expression, thus identifying OPG as a potential diagnostic biomarker for CRC. We also showed that OPG down-regulation was associated with aggressive oncogenic behavior of tumor progression, invasion, and metastasis. Furthermore, reduced OPG expression was an independent predictor of recurrent hepatic metastasis and an independent prognosticator for shorter survival in patients with CRC.

We investigated the regulatory mechanisms for *OPG* gene expression. One possible mechanism that could explain OPG down-regulation was methylation in the gene promoter region [10, 16]. We found treatment with 5-aza-CdR markedly increased *OPG* mRNA expression in the SW620 and HCT 116 cells, which had less than 10% of the mRNA level of CCD 841 CoTr at baseline. Consistent with these findings, 5-aza-CdR treatment restored *OPG* mRNA and protein expression in the CRC cells. These findings indicated that a potential epigenetic mechanism, methylation of the *OPG* promoter, could be involved in repression of the *OPG* gene in CRC cells. We further studied the DNA methylation status of *OPG* promoter using bisulfite pyrosequencing. Down-regulation of OPG occurred in the SW620 and HCT 116 cell lines as a result of enhanced promoter methylation, indicating that aberrant promoter hypermethylation was the cause of *OPG* gene silencing in CRC cells. Similar to these findings, a recent *in vitro* study revealed that the CpG islands of the *OPG* gene are hypermethylated in the human embryonic kidney cell line HEK-293 and osteoblastic cell line HOS-TE85, resulting in lower *OPG* mRNA than in the primary human osteoblastic cell lines hOB and MG-63, both of which have higher *OPG* mRNA levels, but lower methylation [16]. The 5-aza-CdR treatment induced a 20-fold increase in *OPG* mRNA in HEK-293 cells. Lu and colleagues [10] observed reduced OPG expression in nasopharyngeal carcinoma. They found that *OPG* mRNA expression was absent in all 14 nasopharyngeal carcinoma cell lines examined. Furthermore, low OPG protein was discovered in a subset of human carcinoma cell lines established from organs such as the lung, breast, pancreas, liver, prostate, uterine cervix, ovary, and kidney. Consistent with our results, the *OPG* gene was silenced due to hypermethylation of CpG sites in the promoter region.

In addition, we demonstrated the functional role of rOPG in CRC cells. rOPG dose-dependently reduced cell viability, and inhibited MMP-2 and VEGF-A production in HCT 116 cells. This observation was in agreement with previous data showing that OPG is able to reduce cancer cell proliferation in nasopharyngeal carcinoma cells [10]. Another study on osteosarcoma also demonstrated that OPG can prevent tumor cell proliferation and the formation of tumor-induced osteolytic lesions and reduce local tumor growth [17]. Taken together, these results provide new insight into the alterations of OPG expression and activity that are associated with the development and progression of CRC. We suggest that therapeutic targeting of OPG is a potential therapeutic strategy for the treatment of CRC.

In contrast to our results, some previous studies have shown higher expression of OPG in CRC cells [7, 12, 13]. An *in vitro* study reported increased *OPG* mRNA and protein in HT-29 and SW480 cell lines [12]. Another study also reported that 13 CRC cell lines expressed *OPG* mRNA [7]. A recent *in vivo* study showed results similar to those from the *in vitro* studies [13]. Tsukamoto and colleagues [13] showed that tumor tissue samples from 77 CRC patients had significantly higher *OPG* mRNA levels than normal colonic tissue. Also, a CRC patient group with distant metastasis or recurrence exhibited significantly higher *OPG* mRNA levels than the group that did not have distant metastasis or recurrence. Contrary to our results, higher OPG expression was significantly associated with aggressive oncogenic behavior and was identified as an independent prognostic factor for predicting CRC recurrence. These discrepancies could be due to the fact that previous *in vitro* studies did not analyze OPG expression in a normal colonic epithelial cell line for comparison. Previous studies demonstrated production of *OPG* mRNA in CRC cell lines through reverse-transcriptase PCR and an increase in OPG protein concentration that increased over time [7, 12]. However, in these studies, lack of a normal colonic epithelial cell line prevented verification of OPG overexpression in the CRC cell line. Our study included a normal colonic epithelial cell line (CCD 841 CoTr). We also used two primer sets to validate the significant reduction in OPG expression in three CRC cell lines compared to the normal colonic epithelial cell line.

A comparison of OPG expression results in CRC tumor tissue samples in Tsukamoto and colleagues [13] and our study is complicated by many differences in patient characteristics. The survival rate in the Tsukamoto study was over 50%, regardless of OPG expression. We believe that the reason for the higher survival observed in this patient group compared to our study was a smaller proportion of patients with stage IV tumor (7.5%; 48/274) in the previous study than in our study (58.1%; 68/117). Our study group comprised a larger number of patients with advanced CRC. Moreover, in the Tsukamoto study, OPG expression was not detected in normal colonic epithelial cells. Since our study used the same four-tier scoring method as the Tsukamoto study for data interpretation, we assume the primary reason for the difference in results is the use of different antibodies. Other factors that might have influenced OPG detection are differences in the sensitivity of antigen retrieval and staining procedures. Most importantly, previous studies did not present evidence from *in vitro* studies explaining OPG overexpression in CRC. Based on the observed OPG down-regulation in CRC cell lines and the identification of promoter hypermethylation as one of the causes for this down-regulation, we propose that the methylation status of the *OPG* promoter should be analyzed for cancers of various organs with confirmatory reports of OPG expression.

Experimental data on OPG expression conflict in other types of human malignancy. Prostate cancer cells produce and release OPG *in vitro* [9]. The human prostate cancer cell line PC3 produced sufficient OPG to yield significant protection against TRAIL-induced apoptosis. In contrast, in an *in vivo* study, administration of OPG decreased the growth of prostate cancer xenografts in nude mice [18]. Similarly, a previous study on the effect of OPG on prostate cancer burden found that OPG markedly reduced tumor size at bone sites and suppressed progression of established tumor lesions and development of new lesions [14]. Treatment of a murine model of multiple myeloma with recombinant OPG (rOPG) resulted in significantly decreased tumor burden and increased survival [19]. A clinical study demonstrated that OPG was significantly decreased in the serum of patients with multiple myeloma, compared to that of healthy individuals [20]. These data are consistent with our results.

In conclusion, based on our experiments, we suggest that OPG is potentially involved in the regulation of CRC progression. OPG was ubiquitously down-regulated in CRC cell lines. Down-regulation of OPG by promoter hypermethylation may be one mechanism contributing to tumor growth and progression. We demonstrated that reduction in OPG expression was significantly associated with aggressive oncogenic behavior of higher histological grade, presence of nodal and hepatic metastases, occurrence of recurrent hepatic metastasis, advanced stage, and vascular invasion, and was an independent predictor for recurrent hepatic metastasis and an independent prognosticator for poor survival. These results suggest that OPG may be a potential tumor suppressor. Restoration of OPG expression may offer a new therapeutic approach for treating patients with CRC.

## MATERIALS AND METHODS

### Patients and tissue specimens

Tissue samples were obtained from 117 consecutive patients who underwent surgery for primary adenocarcinoma of the colon and rectum. Two independent board-certified pathologists reviewed all hematoxylin and eosin-stained slides and selected the most representative slide from each case for immunohistochemical staining. Clinicopathological data, including age, sex, size of the primary and metastatic tumor, histological grade, pathological tumor stage, the presence of nodal metastasis and/or distant metastasis, local recurrence, TNM stage group, the presence of lymphovascular invasion, multiplicity of the metastatic tumor, and postoperative follow-up, were collected. All tumors were assessed for histological grade according to the World Health Organization classification [21] and were postoperatively staged according to the seventh edition of the American Joint Committee on Cancer staging system [4]. None of the patients underwent preoperative neoadjuvant chemotherapy or neoadjuvant concurrent chemoradiation therapy. Informed consent was obtained from all subjects. This study was reviewed and approved by the institutional review board of Kangbuk Samsung Hospital, Seoul, Republic of Korea (2015-04-053).

### Cell lines and treatments

The human normal colonic epithelial cell line, CCD 841 CoTr, and the CRC cell lines, SW620 and HCT 116, were purchased from the American Type Culture Collection (Manassas, VA, USA) and maintained in Dulbecco's Modified Eagle's Medium (DMEM) or Roswell Park Memorial Institute (RPMI) 1640 medium supplemented with 10% heat-inactivated fetal bovine serum (FBS), penicillin (100 U/mL) and streptomycin (100 μg/mL) (Gibco, Life Technologies, Grand Island, NY, USA). All cell lines were cultured in a humidified atmosphere of 5% CO_2_ at 37°C. The 5-aza-CdR (Sigma-Aldrich, St. Louis, MO, USA) dissolved in dimethyl sulfoxide (DMSO) (Sigma-Aldrich) at 50 mg/mL as a stock solution; this was stored at −20°C. DMSO concentration was 0.001%, and the same concentration was used as vehicle. Immediately before use, stock solutions were diluted in RPMI 1640 without FBS. Native rOPG expressed by mammalian cells was purchased (R & D Systems, Minneapolis, MN, USA).

### cDNA synthesis

RNase-free DNase I treatment was performed to remove contaminating genomic DNA from purified total RNA. Isolated total RNA was diluted to 1 μg/μL with sterile diethylpyrocarbonate (DEPC)-treated H_2_O and 2.5 μL was added to reactions containing 1× DNase I buffer and 1 unit DNase I (final volume, 10 μL). After incubation at 37°C for 30 min, reactions were stopped at 70°C for 10 min. DNase I-treated RNA was reverse-transcribed into first-strand cDNA using random primers. One microgram DNase I-treated RNA and 250 ng random primers were mixed in a 0.5-mL polymerase chain reaction (PCR) tube and brought to 11 μL with sterile DEPC-treated H_2_O, heated at 65°C for 5 min, and chilled quickly on ice. Other reagents were added for a reaction of 20 μL with the indicated final concentrations: 1× First-Strand Buffer, 10 mM DTT, 0.5 mM each dNTP and 200 units Superscript II reverse-transcriptase (Invitrogen, Life Technologies). Reactions were incubated at 42°C for 1 h, heated to 70°C for 10 min and stored at −20°C.

### Quantitative real-time PCR

After reverse transcription, 3 μL was used as a PCR template. PCR was in 10 μL containing 1× SsoFast EvaGreen supermix (Bio-Rad Laboratories, Hercules, CA, USA) and 300 nM each primer. Mixtures were added to 384-well plates for amplification using a CFX Connect Real-Time PCR Detection System (Bio-Rad Laboratories) for 95°C for 10 min, 95°C for 10 s and 60°C for 30 s for 40 cycles. Amplification patterns were analyzed and threshold cycle numbers (C_T_) for each sample were determined using CFX Manager Software (Bio-Rad Laboratories). The ΔΔC_T_ method was used to calculate relative expression of target gene after normalization by C_T_ to GAPDH [22]. Amplification of the target gene was confirmed by melting curve analysis and target amplicon size was confirmed by agarose gel electrophoresis. Each sample was assayed in triplicate.

We used two sets of OPG primer pairs to confirm observed results: OPG set #1, sense: 5′-TTGGTCTCCTG CTAACTCA-3′ and antisense: 5′-GAAGAATGCCTCCT CACAC-3′; OPG set #2, sense: 5′-CAGGCACTTGAGGC TTTC-3′ and antisense: 5′-GGGTTTATTGGAGGAGAT GTTAG-3′; GAPDH, sense: 5′-ACCAGGTGGTCTCCTC TGAC-3′ and antisense: 5′-TGCTGTAGCCAAATTCGTTG-3′.

### Western blot

CCD 841 CoTr, HT-29, SW620 and HCT 116 cells (5 × 10^4^ cells/well) in 6-well plates were incubated at 37°C in 5% CO_2_ in DMEM or RPMI containing 10% FBS. Whole cells lysates were prepared in lysis buffer (50 mM Tris [pH 7.5], 1% NP-40, 150 mM NaCl, 0.5% sodium deoxycholate and 0.1% SDS) containing protease inhibitors (Protease Inhibitor Cocktail Tablet; Roche Applied Science, Mannheim, Germany), and cleared by microcentrifugation (13,000 rpm for 20 min at 4°C). The resulting lysates were assessed for protein concentration, and 20–30 μg of each protein sample was resolved by 12% SDS-PAGE, and electroblotted onto nitrocellulose membranes (GE Healthcare, London, UK). After 1 h incubation in blocking solution (5% non-fat milk in TBST), the membranes were exposed to the appropriate primary antibodies overnight at 4°C. The primary antibodies included: those against OPG (1:200, Abcam, Cambridge, MA, USA), matrix metalloproteinase-2 (MMP-2; 1:1,000, Merck Millipore, Billerica, MA, USA), vascular endothelial growth factor A (VEGF-A; 1:1,000, Merck Millipore) and β-actin (1:5,000, Santa Cruz Biotechology, Santa Cruz, CA, USA). The blots were then washed three times in TBST and incubated with HRP-conjugated secondary antibodies for 1 h at room temperature. The results were visualized using an enhanced chemiluminescence system (Amersham Sciences, Chicago, IL, USA).

### Enzyme-linked immunosorbent assay

For analysis of OPG production, culture media was harvested and centrifuged to remove cellular debris. Media was concentrated by centrifugal filtration at 4,000 rpm for 20 min using the Amicon Ultra-10 K concentrator (Merck Millipore). A commercial enzyme-linked immunosorbent assay (ELISA) kit (USCN Life Science, Wuhan, Hubei, China) was used as described by the manufacturer to measure concentrations of human OPG. Each sample was assayed in triplicate.

### Genomic DNA extraction and bisulfite conversion

Genomic DNA was extracted from cultured cell line using NucleoSpin 96 tissue extraction kits (Macherey-Nagel, Duren, Germany) and quantified using a DropSense96 multichannel spectrophotometer (Trinean, Gentbrugge, Belgium). Bisulfite treatment was performed using the MethylDetector bisulfite modification kit (Active Motif, Carlsbad, CA, USA) on 2 μg of DNA according to the protocols provided by the manufacturer.

### Pyrosequencing

DNA methylation of OPG was determined by bisulfite pyrosequencing. Primers were designed by the Pyrosequencing Assay Design Software, Ver. 1.0.6 (Biotage, Uppsala, Sweden). To ensure distinct pyrosequencing signals, the previously bisulfite-modified DNA (100 ng) was amplified by 45× cycled PCR using the Blend Taq-Plus-(Toyobo, Osaka, Japan) with biotin-labeled primer. PCR products were immobilized to streptavidin sepharose beads via biotin affinity. PCR products were denatured to single-stranded DNA (ssDNA) and annealed with sequencing primers. Complexes of bead-bound ssDNA and primer were applied to a PyroMark pyrosequencer (Biotage) with appropriate reagents. Raw results were analyzed and visualized using Pyro Q-CpG Software, Ver. 1.0.0 (Biotage). Pyrosequencing was performed for three independent bisulfite reactions and average methylation frequency for each CpG site was calculated.

### 3-(4, 5-dimethylthiazol-2-yl)-2, 5-diphenyltetrazolium bromide (MTT) assay

Cell viability was assessed using the MTT assay. Briefly, cells were divided into 96-well plates (100 μL/well) and cultured for 24 h. rOPG at concentrations of 0 to 10 μg/mL was added, and the cells were incubated for an additional 24 h. At the end of the treatment, the cells were washed twice with phosphate-buffered saline (PBS), and the culture medium containing 10% MTT was added. After incubation with MTT at 37°C for 4 h, 100 μL DMSO was added to each well, followed by gently shaking for 10 min to achieve complete dissolution. Cell viability was determined by the differences in absorbance at wavelength of 570 nm. All experiments were performed in triplicate.

### Immunohistochemistry

Formalin-fixed tissue was dehydrated in a graded ethanol series and embedded in paraffin. Paraffin blocks were sectioned at 4 μm on a standard rotary microtome, and slices were brought from a water bath on cleaned slides. OPG protein expression was assessed by immunohistochemistry using the Bond Polymer Intense Detection System (Vision Bio-Systems, Mount Waverley, Victoria, Australia), following the manufacturer's instructions. The general procedure has been described [23–28]: 4-μm sections of formalin-fixed, paraffin-embedded tissue were deparaffinized with Bond Dewax Solution (Vision BioSystems), and an antigen retrieval procedure was performed using Bond ER Solution (Vision BioSystems) for 30 min at 100°C. Endogenous peroxidases were quenched with hydrogen peroxide for 5 min. Sections were incubated for 15 min at ambient temperature with rabbit polyclonal anti-OPG antibody (1:100, Abcam, Cambridge, MA, USA). A biotin-free polymeric horseradish peroxidase-linker antibody conjugate system was used with a Bond-maX automatic slide stainer (Vision BioSystems), and visualization was performed using 1 mM 3, 3-diaminobenzidine (DAB), 50 mM Tris-HCl buffer (pH 7.6) and 0.006% H_2_O_2_. Sections were counterstained with hematoxylin. Slides were dehydrated following a standard procedure and sealed with coverslips. To minimize interassay variation, positive and negative control samples were included in each run. The positive control was normal liver tissue. The negative control was prepared by substituting non-immune serum for the primary antibody; no detectable staining was evident.

Immunohistochemical staining was analyzed by two independent board-certified pathologists. OPG staining intensity was graded as negative (0), weak (1+), moderate (2+) or strong (3+), as described previously [8]. No heterogeneous staining was observed within individual slides and estimation of the proportion of staining was not required. Disagreements between the two pathologists were resolved by consensus.

### Statistical analysis

We used the unpaired Student's *t*-test to compare expression levels of OPG and promoter methylation frequency between CRC and normal colonic tissue samples and cell lines. Chi-square or Fisher's exact tests were performed to determine whether alteration in OPG expression was associated with CRC patient clinicopathological characteristics. Multivariate logistic regression analysis with a backward stepwise elimination method was used to identify independent predictors of recurrent hepatic metastasis. A logistic regression equation indicated the probability of developing recurrent hepatic metastasis based on a combination of independent predictors. Univariate and multivariate survival analyses were used to determine the prognostic implications of OPG expression. Cancer-specific survival was defined as the interval from surgery to death from CRC. Loss to follow-up, death from a cause other than CRC and survival until the end of the follow-up period were considered censoring events. Survival curves were drawn using the Kaplan-Meier method and differences were analyzed by log-rank test for univariate survival analysis. Multivariate survival analysis used the Cox proportional hazard model (95% confidence interval) with a backward stepwise elimination method. All covariates with statistical significance on univariate analysis were entered into multivariate analysis. Least significant covariates were removed from the model by backward stepwise elimination. Statistical analyses used SPSS version 18.0 (IBM SPSS Inc., Chicago, IL, USA). *P*-values less than 0.05 were considered statistically significant.
